# Adenosine Generated by Regulatory T Cells Induces CD8^+^ T Cell Exhaustion in Gastric Cancer through A2aR Pathway

**DOI:** 10.1155/2019/4093214

**Published:** 2019-12-14

**Authors:** Linsen Shi, Min Feng, Shangce Du, Xu Wei, Hu Song, Xu Yixin, Jun Song, Guan Wenxian

**Affiliations:** ^1^Department of Gastrointestinal Surgery, The Affiliated Hospital of Xuzhou Medical University, Xuzhou, China; ^2^The Affiliated Drum Tower Clinical College of Nanjing Medical University, Nanjing, China; ^3^Department of Gastrointestinal Surgery, The Affiliated Drum Tower Hospital of Nanjing Medical University, Nanjing, China

## Abstract

**Background:**

Adenosine, derived from the degradation of ATP via ectonucleotidases CD39 and CD73, is a critical immunosuppressive metabolite in the hypoxic microenvironment of tumor tissue. Adenosine signaling via A2aR can inhibit the antitumor immune response of CD8^+^ T cells. CD39 and CD73 high-expressing Tregs play a critical role in tumor immune evasion of gastric cancer (GC). The present study investigated the underlying mechanism by which Tregs suppress antitumor immune responses in GC.

**Materials and Methods:**

Fifty-two GC samples were collected, and the frequency of FoxP3^+^ Tregs and CD8^+^ T cells and density ratios of A2aR^+^/CD8^+^ T cells, CD39^+^/FoxP3^+^ Tregs, and CD73^+^/FoxP3^+^ Tregs in GC were assessed with multiplex immunofluorescence. The expression of FoxP3 and A2aR in GC tissues was also detected by the immunoblotting assay. We next investigated the relationship between density of FoxP3^+^ Tregs, ratio of A2aR^+^/CD8^+^ T cells, and clinicopathological parameters. At the same time, Tregs and CD8^+^ T cells were isolated from peripheral blood of five GC patients, and the antagonists of CD39 and CD73 were used to assess the ability of Tregs to decompose ATP into adenosine. In addition, we cocultured CD8^+^ T cells and Tregs with antagonists of A_2a_R and A_2b_R in order to examine the alterations in immune function of CD8^+^ T cells.

**Results:**

The density of both FoxP3^+^ Tregs and A2aR^+^/CD8^+^ T cells was higher in GC tissue compared to peritumoral normal tissue and significantly correlated with the TNM stage, lymph node metastasis, and distant metastasis of GC. The process of Treg hydrolysis of ATP into adenosine was blocked by the antagonists of CD39 and CD73. In addition, Tregs could induce apoptosis and inhibit proliferation of CD8^+^ T cells, while this effect could be obviously reduced by applying the antagonist of A_2a_R or A_2a_R^+^A_2b_R. Moreover, IFN-*γ*, TNF-*α*, and perforin generated by CD8^+^ T cells could also be inhibited through the adenosine A2aR pathway.

**Conclusions:**

The FoxP3^+^ Tregs and A2aR^+^/CD8^+^ T cells were excessively infiltrated in GC tissue. Tregs from GC can decompose ATP to adenosine and in turn induce apoptosis and inhibit the proliferation of CD8^+^ T cells through the A2aR pathway, further leading to immune escape of GC.

## 1. Introduction

Gastric cancer (GC) is the third leading cause of cancer-related mortality worldwide and the most prevalent cancer in Eastern Asia [1, 2]. Surgical resection remains the main treatment approach for most patients with GC. The optimal therapeutic strategy, particularly for patients with locally advanced cancer, remains undefined. Recently, immunotherapy has become the most rapidly evolving treatment strategy in oncology. Combinatory approaches with programmed cell death protein 1 (PD-1) and cytotoxic lymphocyte antigen 4 (CTLA-4) immune-checkpoint inhibitors have shown a promising antitumor activity in advanced or metastatic GC [3–5] but the long-term efficacy warranting further verification in more phase 2 and 3 trial studies.

Adenosine, generated from ATP by the ectonucleotidases CD39 and CD73, is a critical immunosuppressive metabolite in the hypoxic microenvironment of tumor tissue [6, 7]. Under stress conditions, such as ischemia, anoxia, trauma, and inflammation, extracellular adenosine concentrations increase 100 times compared to normal levels [8]. Adenosine signaling via A2aR can not only inhibit the antitumor immune response of immune effector cells such as CD8^+^ T cells, NK cells, DC cells, and macrophages but also enhance the proliferation and polarization of immunosuppressive cells, thereby promoting progression of neoplasm [9–11]. Adenosine also decreases tumor-derived extracellular adenosine via respiratory hyperoxia or coinhibition of CD73 where A2aR could improve the antitumor immune responses by enhancing the cytotoxic capacity of CD8^+^ T and natural killer (NK) cells [11–13].

CD4^+^CD25^+^ Treg, which represents about 5% of circulating CD4^+^ T lymphocytes in the human peripheral blood, has an indispensable role for the maintenance of self-tolerance and immune homeostasis [14]. CD39 and CD73 high-expressing Tregs play a critical role in tumor immune evasion [15, 16]. However, the underlying mechanism by which Tregs promote GC development and whether adenosine contributes to the immunosuppressive role of Tregs are still unclear.

In this study, we assessed the frequency of FoxP3^+^ Tregs and CD8^+^ T cells and density ratios of A2aR^+^/CD8^+^ T cells, CD39^+^/FoxP3^+^ Tregs, and CD73^+^/FoxP3^+^ Tregs in 52 GC samples with multiplex immunofluorescence. Tregs and CD8^+^ T cells were isolated from peripheral blood, while antagonists of CD39 and CD73 were used to assess the ability of Tregs to degrade ATP to adenosine. Moreover, we cocultured Treg and CD8^+^ T cells with A_2a_R and A_2b_R antagonists to verify whether Tregs can inhibit the immune function of CD8^+^ T cells through the A2aR pathway.

## 2. Materials and Methods

### 2.1. Patients and Samples

Fifty-two GC patients, who received operations in The Affiliated Hospital of Xuzhou Medical University between December 2015 and November 2016, were enrolled in this study. All patients were confirmed by pathological examination. The clinical stages of tumors were determined according to the TNM classification system of the 7^th^ edition of the American Joint Committee on Cancer. The clinicopathological characteristics of patients are shown in Table 1. Among them, the median age was 61.3 years (range, 31–85 years), and 6 patients had stage I, 17 had stage II, 25 had stage III, and 4 had stage IV tumors. Among 52 patients, 39 of them were diagnosed with adenocarcinoma, 9 with mucinous adenocarcinoma, and 4 with signet-ring cell carcinoma. Tumor and corresponding peritumor tissues (at least 5 cm distant from the tumor site) were obtained from each patient. Peripheral blood (50–60 ml) was collected from five random GC patients.

Patients who received radiochemotherapy, received immunotherapy, suffered from other cancers, or had a history of an autoimmune disease were excluded from this study. Written informed consent was obtained from all the participants. This project was approved by the Ethics Committee of The Affiliated Hospital at Xuzhou Medical University.

### 2.2. Reagents and Antibodies

Isolation kits for CD8^+^ T cells and CD4^+^CD25^+^CD127^low/−^ regulatory T cells and isolation LD and MS columns were purchased from Miltenyi Biotec (Bergisch Gladbach, Germany). Rabbit polyclonal antibody to human A2aR and FoxP3 was obtained from Abcam (Cambridge, USA), while mouse polyclonal antibody to human CD8, CD39, CD73 and human lymphocyte separation solution was acquired from LianKe MultiSciences (Hangzhou, China). ARL67156 (CD39 antagonist) was obtained from Tocris Bioscience (Bristol, UK). *α*,*β*-Methylene-ADP (CD73 antagonist) was obtained from Santa Cruz (Delaware Ave, USA). MRS1754 (A_2b_R antagonist) and ZM241385 (A_2a_R antagonist) were purchased from Sigma (St. Louis, USA). All the antagonists were dissolved in DMSO and had a final concentration less than 3/1000. ATP was dissolved in DMSO and then further diluted in physiological saline. ATP and IFN-*γ* assay kits were acquired from Jiancheng (Nanjing, China). TNF-*α* and perforin assay kits were obtained from KeyGen Biotech (Nanjing, China). The adenosine assay kit was obtained from BioVision (Milpitas, USA). The cAMP assay kit was obtained from Cloud-Clone Corp. (Wuhan, China). The CFSE Cell Proliferation Assay and Tracking Kit was purchased from BestBioScience (Shanghai, China). PE Annexin V Apoptosis Detection Kit was obtained from BD Biosciences (Franklin Lakes, USA).

### 2.3. Multiplex Immunofluorescence

The paraffin-embedded tissue slides were dewaxed and rehydrated and then blocked with PBST/5% BSA for 30 min at room temperature. The sections were incubated with the primary antibody overnight at 4°C. The secondary antibodies (Alexa Fluor 488 goat anti-rabbit IgG (H + L) and Alexa Fluor 539 goat anti-mouse IgG (H + L); Life Technologies, Los Angeles, CA, USA) were used to bind the primary antibodies for 60 min at room temperature. After counterstaining with 4′,6-diamidino-2-phenylindole (DAPI) (P36931; Life technologies) for 10 min, the slides were observed under a high-resolution slide scanner (Pannoramic MIDI; 3DHISTECH, Budapest, Hungary). Positive lymphocytes (Tregs and CD8^+^ T cells), Tregs with CD39^+^/CD73^+^ and CD8^+^ T cells with A2aR^+^, in 5 randomly selected high-power microscopic fields (HPFs, 40x 10) were counted, and the mean number of positively stained lymphocytes and the ratio of double-positive lymphocytes to corresponding lymphocytes per HPF were also calculated.

### 2.4. Immunoblotting Assay

Fresh tissue was lysed in the radioimmunoprecipitation assay buffer (Sigma). Total protein concentrations were detected using a bicinchoninic acid protein assay kit (Beyotime, Shanghai, China). Total protein (20 *μ*g) was separated by 10% SDS-PAGE and transferred to polyvinylidene fluoride membranes (Millipore, Billerica, MA, USA). Then, the membranes were blocked with 10% nonfat milk for 2 h at room temperature. The specific primary antibodies were cultured with the membranes at 4°C overnight. The membranes were incubated with goat anti-rabbit IgG-HRP (1 : 4000; Proteintech) for 2 h at room temperature. Finally, the blots were visualized using the Chemiluminescent Substrate Kit (Thermo Scientific, MA, USA) and the ChemiDoc MP Imaging System (Bio-Rad, CA, USA).

### 2.5. Collection of PBMCs

Blood samples were collected and immediately transferred into sterile heparinized tubes. Peripheral blood mononuclear cells (PBMCs) were isolated from whole blood by Ficoll-Paque density gradient centrifugation. PBMCs were recovered, washed in AIM-V Medium (Invitrogen), counted using trypan blue dye, and immediately used for subsequent experiments.

### 2.6. Separation of Regulatory T Cells (Tregs)

Tregs were separated from PBMCs by using CD4^+^CD25^+^CD127^low/−^ Magnetic Beads Separation System (MACS) according to the manufacturer's instructions. After washing in PBS, the PBMCs were treated with a cocktail of biotinylated antibodies and Anti-Biotin MicroBeads to deplete non-CD4^+^ and CD127 high cells. Then, positive selection was performed on anti-CD25 magnetic beads to obtain the CD4^+^CD25^+^CD127^low/−^ regulatory T cells. Resulting cells were analyzed by FCM dependent on FoxP3. The purity of FoxP3^+^ cell preparations was consistently 97%.

### 2.7. Separation of CD8^+^ T Cells

CD8^+^ T cells were freshly isolated from PBMCs by negative selection using the CD8^+^ T Cell Separation Kit following the manufacturer's instructions. Isolated cells were immediately used for the next experiment.

### 2.8. Cell Culture

Cells were cultured in RPMI 1640 (Gibco, USA) supplemented with 10% fetal bovine serum (Gibco, USA), penicillin (50 units/ml), and streptomycin (50 *μ*g/ml) in a humidified atmosphere containing 5%CO_2_/95% air at 37°C.

### 2.9. ATP Hydrolysis Assay

MACS-sorted CD4^+^CD25^+^ cells (Tregs) (3 × 10^4^/well) were incubated in wells of flat-bottom 96-well plates for 30 min with 250 mm of ARL67156 or 100 *μ*M of *α*,*β*-methylene-ADP or ARL67156 + *α*,*β*-methylene-ADP, a negative control without the Treg and treated with an equal volume of vehicle. Consequently, the cells were incubated with 20 *μ*M of exogenous ATP; the concentration of unhydrolyzed ATP and adenosine synthesized by Tregs in the supernatant was detected 10–100 min after ATP incubation by using ATP and adenosine assay kits according to the manufacturer's instructions, respectively.

### 2.10. CD8^+^ T Cell Apoptosis and Proliferation Assay

Bead-purified peripheral single CD8^+^ T cells were stained with 1.5 *μ*M CFSE and were incubated at 37°C for 15 min. The process was terminated by using an equal amount of fetal calf serum (Gibco, USA). Subsequently, the cells were washed twice with phosphate-buffered saline and then incubated with CFSE-labeled CD8^+^ T cells (10^5^/well) in wells of 6-well plates with Tregs at the ratio of 1 : 1 (the ratio is decided by our preliminary experimental results; data not shown). CD8^+^ T cells cultured in the medium alone were used as control. MRS1754 (200 nM) and ZM241385 (1 *μ*M) were added to CD8^+^ T cells 30 min before adding the Treg. OKT-3 (2 *μ*g/ml), soluble anti-CD28mAb (2 *μ*g/ml; Miltenyi), and IL-2 (150 IU/ml) were added to induce Treg proliferation.

After 5 days of coculture, apoptotic CFSE-stained CD8^+^ T cells were quantified using Annexin V Apoptosis Detection Kit. In brief, the total cells were washed twice with PBS, resuspended in 500 *μ*l binding buffer, incubated with 5 *μ*l PE-conjugated annexin V and 5 *μ*l APC-conjugated PI for 10 min on ice in the dark, and then analyzed by flow cytometry. Flow cytometry was performed using a BD flow cytometer (BD, USA) equipped with Expo32 software (Beckman Coulter). At the same time, the total cells were washed twice with PBS and resuspended in 500 *μ*l PBS. Then, the proliferation index of CFSE-stained CD8^+^ T cells was calculated using flow cytometry with ModFit software (Topsham, USA), based on the reduction of cell CFSE fluorescence intensity.

### 2.11. cAMP and Cytokine Production Assay

After 5 days of culture, the cell culture supernatant was isolated and the concentration of cAMP, IFN-*γ*, TNF-*α*, and perforin secreted by CD8^+^ T cells was assessed with the ELISA kit according to the manufacturer's instructions.

### 2.12. Statistical Analysis

Statistical analysis was conducted using SPSS 16.0 for Windows (SPSS, Chicago, IL, USA). All numerical data are presented as the mean value ± SEM. The statistical significance of differences between two groups was determined by Student's *t*-test. For multigroup data analysis, an ANOVA was used. All experiments were repeated at least three times independently. A difference was considered significant at *P* < 0.05.

## 3. Results

### 3.1. Number of FoxP3^+^ Tregs and CD8^+^ T Cells and Density Ratios of A2aR^+^/CD8^+^ T Cells, CD39^+^/FoxP3^+^ Tregs, and CD73^+^/FoxP3^+^ Tregs in GC and the Association with Clinicopathological Parameters

We initially compared the densities of CD8^+^ T cells and FoxP3^+^ Tregs between the GC tissues and the paired adjacent normal tissues by multiplex immunofluorescence. We found that the infiltration density of FoxP3^+^ Tregs was significantly higher in cancer tissue (*P*=0.024). CD8^+^ T cells were mildly increased in cancer tissue, while there was no statistical significance (*P*=0.752) compared with peritumoral normal tissue (Figures 1(a) and 1(b)). Then, we evaluated the ratios of A2aR^+^/CD8^+^ T cells, CD39^+^/FoxP3^+^ Tregs, and CD73^+^/FoxP3^+^ Tregs in GC tissues. It was found that the A2aR^+^/CD8^+^ T cell ratio was significantly higher in GC tissues compared with adjacent normal tissues. Similarly, although the ratios of CD39^+^/FoxP3^+^ Tregs and CD73^+^/FoxP3^+^ Tregs in GC tissues were slightly higher compared with controls, no statistical significance was found (Figures 1(a) and 1(c)). Meanwhile, the protein levels of A2aR and FoxP3 in GC tissues and controls were determined by the immunoblotting assay (Figure 1(d)). It was found that the expression of A2aR and FoxP3 was both increased in GC tissues compared with adjacent normal tissues.

To clarify the clinical significance of intratumoral FoxP3^+^ Tregs and A2aR^+^CD8^+^ T cells, we analyzed the possible correlation of these cells with clinicopathological parameters. We found that the frequency of intratumoral FoxP3^+^ Tregs and A2aR^+^CD8^+^ T cells was tightly correlated with the TNM stage (*P*=0.025 and 0.003), lymph node metastasis (*P*=0.046 and 0.025), and distant metastasis (*P*=0.015 and 0.020). No significant correlation was found in other clinicopathological parameters (Table 1). These results suggest that the accumulation of FoxP3^+^ Tregs and A2aR^+^CD8^+^ T cells in tumor tissues should be associated with the progression of GC.

### 3.2. Tregs from GC Patients Decomposed ATP into Adenosine

To identify the role of Tregs from GC patients in adenosine synthesis, Tregs were isolated from patients' PBMCs and then incubated with exogenous ATP. The detailed methods are described in Materials and Methods. It was found that ATP was gradually hydrolyzed from 10 min to 100 min after the setting; while it was cocultured with ARL67156 or *α*,*β*-methylene-ADP (CD39 antagonist) or ARL67156 + *α*,*β*-methylene-ADP (CD73 antagonist), the hydrolysis process was suppressed (*P* < 0.05 vs Tregs) (Figure 2(a)). Meanwhile, the concentration of adenosine was decreased after treatment of ARL67156 or *α*,*β*-methylene-ADP or ARL67156 + *α*,*β*-methylene-ADP (Figure 2(b)). These findings demonstrated that Tregs played a critical role in adenosine synthesis from ATP.

### 3.3. Adenosine Synthesized by Tregs Promoted Apoptosis and Suppressed Proliferation of CD8^+^ T Cells

The in vitro coculture assay was performed to investigate the effect of adenosine synthesized by Tregs on proliferation and apoptosis of CD8^+^ T cells. We found that Tregs promoted apoptosis and suppressed proliferation of CD8^+^ T cells (40.81 ± 6.65%, 1.62 ± 0.25%), while these effects were suppressed with treatment of the antagonist of A_2a_R (17.74 ± 2.20%, 3.27 ± 0.43%, *P*=0.030 and 0.029 < 0.05 vs Tregs) or A_2a_R^+^A_2b_R (9.57 ± 2.33%, 4.02 ± 0.51%, *P*=0.014 and 0.003 < 0.05 vs Tregs) (Figures 3(a)–3(c)). However, the treatment of A_2b_R antagonists alone had no significant suppressive effect (25.72 ± 6.50%, 1.78 ± 0.19%) (P=0.180 and 0.509 > .05 vs Tregs). These results suggested that the effect of Tregs on CD8^+^ T cells was dependent on adenosine A2aR mainly.

### 3.4. Tregs Reduced CD8^+^ T Cell Activity by Promoting cAMP Synthesis

To investigate the underlying mechanism of the suppressive effect of Tregs on CD8^+^ T cells, we determined the level of cAMP derived from the CD8^+^ T cell. It was found that Tregs promoted cAMP expression in CD8^+^ T cells (21.90 ± 1.57 nM). Meanwhile, the treatment of the antagonist of A_2a_R or A_2a_R^+^A_2b_R significantly reduced the concentration of cAMP in conditioned media (15.13 ± 0.89, 13.91 ± 0.82 nM, *P*=0.006 and 0.002 < 0.05 vs Tregs). However, the treatment of the antagonist of A_2b_R had no significant effect on cAMP expression (16.98 ± 1.34 nM) (*P*=0.314 vs Tregs) (Figure 4(a)).

### 3.5. A2aR Tregs Inhibited the Immune Function of CD8^+^ T Cells through A2aR Pathway

The expression of IFN-*γ*, TNF-*α*, and perforin was determined in CD8^+^ T cells. It was found that the IFN-*γ* level was increased significantly with the treatment of ZM241385 (725.70 ± 65.48 pg/ml) or ZM241385 + MRS1754 (779.53 ± 48.72) compared with the Treg treatment alone (405.80 ± 47.92 pg/ml) (*P*= 0.004 and 0.006 < 0.05 vs Tregs) (Figure 4(b)), while MRS1754 treatment alone had no significant effect on IFN-*γ* expression (566.81 ± 52.33 pg/ml) (*P*=0.13 vs Tregs). The levels of perforin and TNF-*α* were also increased remarkably with ZM24138 or ZM241385 + MRS1754 treatment, compared with control (*P* < 0.05 vs Tregs) (Figures 4(c) and 4(d)). These data indicated that adenosine which was increased by Tregs suppressed the immunoactivity of CD8^+^ T cells dependent on the A2aR signaling pathway.

## 4. Discussion

It is well known that the hypoxic and adenosine-rich tumor microenvironment (TME) hampers the body's antitumor immunity [10]. CD39 and CD73 are upregulated in various cell types within the tumor microenvironment, including regulatory T cells (Tregs), stromal cells, and tumor cells [17]. When cells are deprived of nutrients or oxygen, they are driven to break down the extracellular ATP into adenosine [18]. While intracellular adenosine is involved in energy metabolism, nucleic acid metabolism, and the methionine cycle, the extracellular adenosine has an important role in immunoregulation [19].

In the context of cancer, the accumulation of extracellular adenosine can bind to its ligands, especially A2aR, to suppress antitumor immune responses [20, 21]. Stimulation of intracellular adenylyl cyclase caused by A2aR can lead to an increase in intracellular cAMP concentration. Furthermore, the accumulation of intracellular cAMP induces protein kinase A-mediated phosphorylation and activation of COOH-terminal Src kinase (Csk) [22]. Csk may then phosphorylate and inhibit Lck, producing a broad range of immunosuppressive effects, such as diminishing the active immune cytokines (e.g., IFN-*γ*), increasing the production of immunosuppressive cytokines (e.g., TGF-beta and IL-10), and upregulating the alternate immune-checkpoint pathway receptors (e.g., PD-1 and LAG-3) [23].

Here, we found more FoxP3^+^ Treg infiltration in the tumors than in paired adjacent normal tissues, whereas no significance was observed with the frequency of CD8^+^ T cells, similar to the results of other research [24, 25]. At the same time, an increased expression of A2aR on GC tissue infiltrating CD8^+^ T cells was observed, but the density ratios of CD39^+^/FoxP3^+^ Tregs and CD73^+^/FoxP3^+^ Tregs had no significant difference. Previous studies have shown that Tregs from cancer patients expressed high levels of CD39, as a rate-determining step in the generation of immunosuppressive adenosine [26, 27]. The reason for these contradictory findings may be attributable to heterogeneity of the tumor and the bias caused by the relatively small number of cases included in this study. The higher frequency of FoxP3^+^ Tregs and density ratios of A2aR/CD8^+^ T cells in GC tissue were also correlated with the cancer stage, lymph node metastasis, and distant metastasis. Furthermore, we demonstrated that Tregs from GC patients could decompose ATP to adenosine. This process was blocked by ARL67156 and *α*,*β*-methylene-ADP, which are antagonists of CD39 and CD73. This indicates that the Treg and adenosine may be involved in the immune escape of GC, and the Treg could be one of the important sources of adenosine in the immunosuppressive TME of GC.

Nonetheless, the specific mechanisms of Tregs involved in the immune regulation of GC remain unclear, just as the way through which adenosine leads to inactivation of tumor immune effector cells (CD8^+^ T, NK, etc.). Consequently, we cocultured CD8^+^ T and Treg cells from the GC patients, and we found that Tregs could induce apoptosis and inhibit the proliferation of CD8^+^ T cells. Nonetheless, this function was reversed by the antagonists of adenosine receptors, especially A2aR. Furthermore, we detected cAMP, IFN-*γ*, perforin, and TNF-*α* synthesized by CD8^+^ T cells in the culture medium, two of which had elevated concentrations. Based on the above referenced research, it is possible to conclude that adenosine generated by Tregs in GC may lead to increased cAMP synthesis in CD8^+^ T cells and cause its inactivation (decreased IFN-*γ*, perforin, and TNF-*α*) by binding to A2aR.

The adenosine pathway is one of the major inhibitory pathways operating in the TME [28]. Previous studies have indicated that large amounts of adenosine accumulated in the hypoxic TME contribute to suppressing the immune response and promoting tumor progression [29–31]. According to Öztürk et al. [32], aqueous extracts from *S. marianum* can inhibit ADA in gastric cancerous tissues and may have an important role in the immune regulation of GC. Likewise, Ma and colleagues have also found that STO-609 may inhibit the growth of GC through adenosine monophosphate-activated protein kinase [33].

Improvements in systemic therapy for GC have suggested that immunotherapy may be helpful for some patients with gastroesophageal cancer [34]. Nevertheless, achieving durable and reliable curative effects remains a great challenge. As adenosine has a pivotal role in the hypoxia-induced metabolic and immunological TME, several preclinical studies have indicated that the components targeted with antibodies, pharmacologic inhibitors, or siRNAs may suppress tumor progression and metastases [28, 35, 36]. Accordingly, we can speculate that adenosine is also involved in GC and that it may be a potential therapeutic target alone or in combination with existing conventional therapies.

To the best of our knowledge, this is one of the most comprehensive studies on the role of adenosine and Tregs in immunoregulation of GC. Nevertheless, several limitations in the present study do exist: First, this study can be defined as a preliminary study due to the sample size that was not large enough and due to the lack of healthy donors, and thus, more research is necessary to further verify our results. Second, many other factors such as IFN-*γ*^+^ Th1 response, CTLA-4, and LAG3-mediated effector T cell exhaustion are all involved in Treg-mediated tumor immune escape, which means that it is not possible to completely exclude the interference of other confounding factors on the results.

In conclusion, the present data indicate that accumulation of Tregs in GC can decompose ATP to adenosine and then induce apoptosis and inhibit the proliferation of CD8^+^ T cells, leading to immune inactivation and evasion that mainly occur through the A2aR pathway. The adenosine A2aR pathway may be a promising therapeutic target for gastric cancer. Further studies with specific mechanisms of the adenosine pathway in gastric cancer and in vivo experimental studies are necessary to further verify these findings.

## Figures and Tables

**Figure 1:** Expression status of A2aR on CD8^+^ T cells and CD39 and CD73 on FoxP3^+^ Tregs in GC tissue. (a) Representative images of A2aR on CD8^+^ T cells and CD39 and CD73 on FoxP3^+^ Tregs, stained by 3-color tissue immunofluorescence in paired GC tissues. A2aR and FoxP3^+^ Tregs were visualized using the Cy3 channel (red), and CD8^+^ T cells and CD39 and CD73 were visualized using the FITC channel (green). DAPI was used to visualize nuclei (blue). Scale bars = 50 *µ*m in all images. (b) Densities of CD8^+^ T cells and FoxP3^+^ Tregs and (c) ratios of A2aR^+^/CD8^+^ T cells, CD39^+^/FoxP3^+^ Tregs, and CD73^+^/FoxP3^+^ Tregs were also compared. (d) Representative images of A2aR and FoxP3 in 5 paired GC tissues by immunoblotting assays. T: cancer tissue; N: peritumoral normal tissue; n.s.: no statistical significance. ^*∗*^*P* < 0.05; ^*∗∗*^*P* < 0.01.

**Figure 2:** Antagonists of ectonucleotidases CD39 and CD73 affect the activity of Tregs to synthesize adenosine from ATP. (a) Tregs (3 × 10^4^/well) were incubated in 96-well plates for 30 min with vehicle (DMSO), 250 *μ*Μ ARL67156 (CD39 antagonist), *α*,*β*-methylene-ADP (CD73 antagonist) (100 *μ*M), or ARL67156 + *α*,*β*-methylene-ADP, a negative control without the Treg and treated with an equal volume of vehicle. Then, exogenous ATP (20 *μ*M) was added, and the concentration of unhydrolyzed ATP was detected 10 to 100 min after treatment (^*∗*^*P* < 0.05, ^*∗∗*^*P* < 0.01, and ^*∗∗∗*^*P* < 0.001 vs Tregs). (b) The concentration of adenosine was also detected 10 to 100 min after treatment (^*∗*^*P* < 0.05, ^*∗∗*^*P* < 0.01, and ^*∗∗∗*^*P* < 0.001 vs Tregs). In ANOVA, all experiments are repeated at least five times.

**Figure 3:** Treg induces apoptosis and inhibits proliferation of CD8^+^ T cells. (a, b) Bead-purified peripheral single CD8^+^ T cells were stained with 1.5 *μ*M CFSE and incubated at 37°C for 15 min. Subsequently, the cells were washed twice with phosphate-buffered saline. CFSE-labeled CD8^+^ T cells (10^5^ cells/well) were incubated in 6-well plates with Tregs at the ratio of 1 : 1; MRS1754 (A_2b_R antagonist; 200 nM) and ZM241385 (A_2a_R antagonist; 1 *μ*M) were added to CD8^+^ T cells 30 min before adding Tregs. CD8^+^ T cells without Treg coculture and treated with vehicle were set as control. OKT-3 (2 *μ*g/ml), soluble anti-CD28mAb (2 *μ*g/ml; Miltenyi), and IL-2 (150 IU/ml) were added to induce Treg proliferation. After 5 days of coculturing, apoptotic CFSE-stained CD8^+^ T cells were quantified using Annexin V Apoptosis Detection Kit. (c) The cell proliferation index of CFSE-stained CD8^+^ T cells was calculated based on the reduction of CFSE-positive cells (^*∗*^*P* < 0.05, ^*∗∗*^*P* < 0.01, and ^*∗∗∗*^*P* < 0.001 vs Tregs). In ANOVA, all experiments are repeated at least five times.

**Figure 4:** Treg inhibits CD8^+^ T cell function by promoting cAMP synthesis. Bead-purified peripheral single CD8^+^ T cells (10^5^ cells/well) were incubated in 6-well plates with Tregs at the ratio of 1 : 1. MRS1754 (A_2b_R antagonist; 200 nM) and ZM241385 (A_2a_R antagonist; 1 *μ*M) were added to CD8^+^ T cells 30 min before adding Tregs. CD8^+^ T cells without Treg coculture and treated with vehicle were set as control. After 5 days of culturing, cAMP (a), IFN-*γ* (b), perforin (c), and TNF-*α* (d) synthesized by CD8^+^ T cells were detected by using ELISA kits according to the manufacturer's instructions (^*∗*^*P* < 0.05, ^*∗∗*^*P* < 0.01, and ^*∗∗∗*^*P* < 0.001 vs Tregs). In ANOVA, all experiments are repeated at least five times.

**Table 1:** Frequency of FoxP3^+^ Tregs and density ratios of A2aR^+^/CD8^+^ T cells in GC tissues according to clinicopathological parameters.

Variables	*n* = 52	FoxP3^+^ (cells/HPF)	*P* value	A2aR^+^/CD8^+^ (%)	*P* value
*Gender*			0.155		0.250
Male	39	18.96 ± 0.68		25.37 ± 1.07	
Female	13	20.86 ± 1.08		22.66 ± 2.16	

*Age, years*			0.152		0.266
≥60	31	20.51 ± 1.00		26.09 ± 1.68	
<60	21	18.81 ± 0.81		23.91 ± 1.14	

*Differentiation*			0.072		0.227
Low	26	18.12 ± 0.75		25.37 ± 1.46	
Medium	15	20.59 ± 1.17		22.34 ± 1.54	
High	11	20.98 ± 1.31		26.77 ± 2.04	

*Stage (TNM)*			0.025^*∗*^		0.003^*∗*^
I-II	23	17.48 ± 0.81		21.61 ± 1.36	
III-IV	29	20.99 ± 0.80		27.31 ± 1.31	

*Lymphatic metastasis*			0.003^*∗*^		0.025^*∗*^
Negative	16	16.85 ± 0.97		23.17 ± 1.48	
Positive	36	20.58 ± 0.70		28.12 ± 1.25	

*Distant metastasis*			0.015^*∗*^		0.020^*∗*^
Negative	48	19.06 ± 1.12		22.72 ± 1.74	
Positive	4	23.47 ± 1.52		29.38 ± 2.15	

*Classification*			0.527		0.258
Adenocarcinoma	39	19.10 ± 0.66		23.92 ± 1.11	
Mucinous adenocarcinoma	4	21.35 ± 2.44		25.93 ± 3.47	
Signet-ring cell carcinoma	9	20.04 ± 1.41		28.05 ± 2.30	

^*∗*^ *P* < 0.05.

## Data Availability

All the data used to support the findings of this study are included within the article.
